# Application Value Analysis of Seven-Autoantibody Panel in the Lung Cancer Screening in Yunnan

This article has been retracted.

**DOI:** 10.1155/2022/2368155

**Published:** 2022-07-04

**Authors:** Wenrun Li, Yi Sun, Ning Xu

**Affiliations:** Department of Medical Laboratory, The First People's Hospital of Yunnan Province, The Affiliated Hospital of Kunming University of Science and Technology, Kunming, Yunnan, China

## Abstract

**Objective:**

To study the application value of seven-autoantibody (anti-CAGE, anti-GAGE7, anti-GBU4-5, anti-MAGE A1, anti-P53, and anti-PGP9.5, anti-SOX2) in lung cancer (LC) screening in Yunnan.

**Methods:**

The clinical data of 329 lung cancer patients and 202 nonlung cancer controls in the First People's Hospital of Yunnan Province from November 2018 to April 2022 were retrospectively analyzed. The detection results of anti-CAGE, anti-GAGE7, anti-GBU4-5, anti-MAGE A1, anti-P53, anti-PGP9.5, and anti-SOX2 were collected. The receiver operating curve (ROC) was used to analyze the value of these seven-autoantibody in the detection of LC alone and in combination, and the area under the curve (AUC), sensitivity, specificity, and cut-off values were calculated.

**Results:**

The levels of anti-CAGE, anti-GAGE7, anti-GBU4-5, anti-MAGE A1, anti-P53, anti-PGP9.5 and anti-SOX2 in LC patients were significantly higher than those in the controls, and the differences were statistically significant (*P* < 0.001). The AUC of anti-CAGE, anti-GAGE7, anti-GBU4-5, anti-MAGE A1, anti-P53, anti-PGP9.5, and anti-SOX2 for the diagnosis of LC were 0.586 (95% CI: 0.537–0.634, *P* < 0.001), 0.620 (95% CI: 0.572–0.667, *P* < 0.001), 0.570 (95% CI: 0.521–0.619, *P*=0.007), 0.612 (95% CI: 0.563–0.660, *P* < 0.007) 0.001), 0.561 (95% CI: 0.510–0.611, *P*=0.019), 0.667 (95% CI: 0.619–0.715, *P* < 0.001), 0.587 (95% CI: 0.538–0.636, *P* < 0.001), respectively. The AUC of combined detection of LC was 0.719 (95% CI: 0.676–0.761, *P* < 0.001). The positive rate of the combined detection of seven-autoantibody in the LC group was 48.02% (158/329), which was significantly higher than that of the control group (13.86% (28/202)), the difference was statistically significant (*χ*^2^ = 64.183, *P* < 0.001).

**Conclusion:**

The individual detection and combined detection of the seven-autoantibody have a certain value in the diagnosis of LC in Yunnan, and it can provide a certain reference for clinical LC screening.

## 1. Introduction

Lung cancer (LC) is currently one of the most common malignancies and the leading cause of cancer-related deaths worldwide [1, 2]. The 5-year average survival rate of LC is only 17.4%, and with the development of the tumor, the survival rate will further decrease [3]. Although the 10-year survival rate of stage Ia LC patients is 92%, 85% of LC patients are diagnosed at an advanced stage and lose the opportunity for surgery, so early detection and treatment are of great significance for improving the overall survival rate of LC patients [3, 4].

Although serum tumor markers have a certain predictive value for LC, they are mainly used for the detection of curative effects and have low diagnostic value for LC [5, 6]. The overexpression, mutation, and folding of tumor-associated antigens can activate the body's immune system to produce corresponding autoantibodies, which are called tumor-associated autoantibodies (TAABs), and such TAABs can persist in peripheral blood for a long time and can be detected 5 years before the positive CT scan in the asymptomatic stage of LC [7]. TAABs currently have good diagnostic performance in the early diagnosis of LC. For example, Ouyang et al. [8] found that the combined detection of seven-autoantibody has important value in the early screening of LC. Wang et al. [9] confirmed that anti-GNA11 has the potential to be a new serological marker for the diagnosis of esophageal squamous cell carcinoma.

In this study, we evaluated the efficacy and value of seven-autoantibody (anti-CAGE, anti-GAGE7, anti-GBU4-5, anti-MAGE A1, anti-P53, anti-PGP9.5, and anti-SOX2) in the diagnosis of LC in Yunnan Province.

## 2. Materials and Methods

### 2.1. Subjects

A total of 329 LC patients admitted to the First People's Hospital of Yunnan Province from November 2018 to April 2022 was 155 males and 174 females. The average age was (49.49 ± 12.03) years old. All LC patients were diagnosed by histopathological examination, including 125 cases of lung squamous cell carcinoma, 143 cases of lung adenocarcinoma, and 61 cases of small cell lung cancer. According to TNM staging criteria, 89 cases were in stage I, 95 in stage II, 73 in stage III, and 72 in stage IV. The diagnostic criteria for LC were based on the Chinese Medical Association guidelines for clinical diagnosis and treatment of lung cancer (2018 Edition) [10]. Inclusion criteria: (1) the LC patients were newly diagnosed, without surgery, radiotherapy and chemotherapy; (2) histopathologically diagnosed as LC by biopsy; (3) the clinical stage of the tumor was not clear. At the same time, 202 nonlung cancer controls in our hospital during the same period were collected, including patients with interstitial lung disease, chronic obstructive pulmonary disease (COPD), or asthma. In the control group, there were 105 males and 97 females, with an average age of (50.65 ± 12.51) years.

## 3. Methods

A total of 4 ml of fasting venous blood was collected from the LC patients and the controls, centrifuged at 2500 r/min for 10 min, then separated the serum, and detected within 8 hours. The samples were detected by an enzyme-linked immunosorbent assay (ELISA) kit (Hangzhou Kaibao Biotechnology Co., Ltd., Hangzhou, China), and the absorbance was read at 450 nm. All the operations were performed in strict accordance with the reagent instructions. The cut-off values of the 7-TAAB kit were: CAGE 7.2 U/ml, GAGE7 14.4 U/ml, GBU4-5 7.0 U/ml, MAGE A1 11.9 U/ml, P53 13.1 U/ml, PGP9.5 11.1 U/ml, SOX2 10.3 U/ml. The experimental procedure of this study was shown in Figure 1.

### 3.1. Statistical Analysis

The SPSS 22.0 software (Armonk, NY, USA) was used for statistical analysis. The detection results of seven-autoantibody (anti-CAGE, anti-GAGE7, anti-GBU4-5, anti-MAGE A1, anti-P53, anti-PGP9.5, anti-SOX2) levels were first tested for normality. The skewed distribution date were expressed as the median (interquartile range). The Mann–Whitney *U* test was used to compare the differences between the two groups. The diagnostic value of seven-autoantibody (anti-CAGE, anti-GAGE7, anti-GBU4-5, anti-MAGE A1, anti-P53, anti-PGP9.5, anti-SOX2) single and combined detection in LC were comprehensively evaluated by receiver operating curve (ROC), and the area under the curve (AUC), sensitivity, specificity, and cut-off value were calculated. The combined detection of serum seven-autoantibody adopted the parallel test (any index of serum 7-TAAB higher than the cut-off value was judged as positive, and if all antibody levels were negative, it was negative). *P* < 0.05 indicated a significant difference.

## 4. Results

### 4.1. Comparison of Clinical Data

The clinical data of the LC patients and the controls were compared, and the results are shown in Table 1. Among the 329 LC patients, the age ranged from 19 to 86 years, with an average age of (49.49 ± 12.03) years, including 155 males and 174 females. Histological typing showed that 125 were squamous cell carcinomas, 143 were adenocarcinomas, and 61 were small cell lung cancers. Among the 202 subjects in the control group, the age ranged from 19 to 82 years, with an average age of (50.65 ± 12.51) years, including 105 males and 97 females. Statistical analysis showed that there were no significant differences in age and sex between the LC patients and the controls (*P* > 0.05).

### 4.2. Comparison of Serum Levels of Seven Autoantibodies in LC Patients and Control Subjects

Comparison of serum levels of seven-autoantibody (anti-CAGE, anti-GAGE7, anti-GBU4-5, anti-MAGE A1, anti-P53, anti-PGP9.5, and anti-SOX2) between LC patients and controls are shown in Table 2. Statistical analysis showed that the levels of anti-CAGE, anti-GAGE7, anti-GBU4-5, anti-MAGE A1, anti-P53, anti-PGP9.5, and Anti-SOX2 in LC patients were significantly higher than those in the controls, the differences were statistically significant (*P* < 0.001).

### 4.3. Analysis of the Value of Serum Seven-Autoantibody and Combined Detection in the Diagnosis of LC

We plotted the receiver operating curve (ROC) of the detection of serum seven-autoantibody (anti-CAGE, anti-GAGE7, anti-GBU4-5, anti-MAGE A1, anti-P53, anti-PGP9.5, and anti-SOX2) alone and in combined detection for LC. The analysis results showed that the serum seven-autoantibody (anti-CAGE, anti-GAGE7, anti-GBU4-5, anti-MAGE A1, anti-P53, anti-PGP9.5, and anti-SOX2) alone had certain diagnostic value in the diagnostic single indicator (Table 3). The AUC of anti-CAGE in the diagnosis of LC was 0.586 (95% CI: 0.537–0.634, *P* < 0.001), the sensitivity was 98.02%, the specificity was only 16.41%, and the cut-off value was 1.850U/mL (Figure 2(a)). The AUC of anti-GAGE7 for the diagnosis of LC was 0.620 (95% CI: 0.572–0.667, *P* < 0.001), the sensitivity was 67.33%, the specificity was 52.28%, and the cut-off value was 1.350 U/mL (Figure 2(b)). The AUC of anti-GBU4-5 for the diagnosis of LC was 0.570 (95% CI: 0.521–0.619, *P*=0.007), the sensitivity was 96.53%, the specificity was only 15.50%, and the cut-off value was 5.050 U/mL (Figure 2(c)). The AUC of anti-MAGE A1 for the diagnosis of LC was 0.612 (95% CI: 0.563–0.660, *P* < 0.001). The sensitivity was 68.32%, the specificity was 47.42%, and the cut-off value was 0.150 U/mL (Figure 2(d)). The AUC of anti-P53 for the diagnosis of LC was 0.561 (95% CI: 0.510–0.611, *P*=0.019), the sensitivity was only 46.53%, the specificity was only 64.44%, and the cut-off value was 0.950 U/mL (Figure 2(e)). The AUC of anti-PGP9.5 for the diagnosis of LC was 0.667 (95% CI: 0.619–0.715, *P* < 0.001), the sensitivity was 55.94%, the specificity was 71.43%, and the cut-off value was 0.250 U/mL (Figure 2(f)). The AUC of anti-SOX2 for the diagnosis of LC was 0.587 (95% CI: 0.538–0.636, *P* < 0.001), the sensitivity was 54.46%, the specificity was only 60.79%, and the cut-off value was 0.550 U/mL (Figure 2(g)). The AUC for the combined detection of LC was 0.719 (95% CI: 0.676–0.761, *P* < 0.001), with a sensitivity of 86.14% and a specificity of 48.02% (Figure 2(h)).

### 4.4. Analysis of the Value of Combined Detection of Serum Seven-autoantibody in the Diagnosis of Different Histological Types of LC

We further analyzed the ROC of serum seven-autoantibody in the diagnosis of different histological types of LC, and the results showed that the AUC of serum anti-CAGE, anti-GAGE7, anti-GBU4-5, anti-MAGE A1, anti-P53, anti-PGP9.5, and anti-SOX2 for the diagnosis of squamous cell carcinoma was 0.640 (95% CI: 0.576–0.705, *P* < 0.001) (Figure 3(a)). The AUC for the combined detection of adenocarcinoma was 0.734 (95% CI: 0.680–0.787, *P* < 0.001) (Figure 3(b)). The AUC of combined detection for the diagnosis of small cell lung cancer was 0.717 (95% CI: 0.638–0.796, *P* < 0.001) (Figure 3(c)).

### 4.5. Positive Rate of Combined Detection of Serum Seven-Autoantibody

The positive rate of the combined detection of seven-autoantibody in the LC patients was 48.02% (158/329), which was significantly higher than that of the controls (13.86% (28/202)), the difference was statistically significant (*χ*^2^ = 64.183, *P* < 0.001).

## 5. Discussion

Early diagnosis and treatment before tumor metastasis can significantly improve patient survival. The classic tumor markers in serum have low sensitivity and low specificity in the diagnosis of LC, which cannot fully meet the needs of clinical diagnosis [11]. CT screening can detect small tumors, but CT screening has a high false-positive rate and cannot identify benign and malignant tumors. It is urgent to seek a simple biomarker as a diagnostic tool for LC to reduce the misdiagnosis rate [12]. In the early stage of tumor onset, tumor-associated antigens cause the body to produce an autoimmune response due to gene mutations, protein abnormalities, etc., and stimulate B cells to secrete TAAB. A small amount of tumor-associated antigens produces a large amount of TAAB through the signal amplification of humoral immunity [12–15], and TAAB can be detected several years before clinical symptoms appear, so the detection of TAAB can open up a new way for the early diagnosis of LC.

Cancer associated gene (CAGE), G antigen 7 (GAGE7), RNA helicase autoantibodies GBU4-5 (GBU4-5), and melanoma antigen A1 (MAGE-A1) are all tumor-testis antigens, which are specifically expressed in a variety of malignant tumors and their levels are higher in LC patients [16, 17]. P53 is a tumor suppressor that activates the DNA repair pathway and inhibits the proliferation of tumor cells. It can appear before the clinical diagnosis of LC [18, 19]. Protein gene product 9.5 (PGP9.5) is pantothenate hydrolase, a biomarker for non-small-cell lung cancer [20, 21]. SRY-box containing gene 2 (SOX2) is a transcription factor that is expressed in LC, breast cancer, and other malignant tumor tissues, and the ability of cancer cells to metastasize to distant sites is proportional to its overexpression [22]. The autoantibodies selected in this study may also exist in other cancer patients. For example, the production of P53 antibody is closely related to the occurrence of various cancers [18], SOX2 antibody can be found in liver cancer [23], PGP9.5 antibody can be found in colorectal cancer [20], and MAGE-A has been confirmed to be highly correlated with LC [22].

The results of this study showed that the serum levels of seven-autoantibody in LC patients were significantly higher than those in controls, which was consistent with the research results of Chapman et al. [24], indicating that the levels of each autoantibody in the serum of nonlung cancer patients were lower; therefore, we can easily distinguish lung cancer patients and nonlung cancer patients. After analyzed by ROC, we found that the AUCs of anti-CAGE, anti-GAGE7, anti-GBU4-5, anti-MAGE A1, anti-P53, anti-PGP9.5, and anti-SOX2 for the diagnosis of LC were all higher than 0.5. Therefore, we judged that the detection of serum levels of seven-autoantibody has application value in the diagnosis of LC, and the combined detection AUC was higher, which was 0.719, and the sensitivity was as high as 86.14%, but the specificity was only 48.02%. The positive rate of the combined detection of seven-autoantibody in the LC group was also significantly higher than that of the controls, indicating that the combined detection of seven-autoantibody cannot be used as an independent diagnostic method for lung cancer but can be used as an auxiliary method because its specificity is too low. At present, researchers have paid attention to the value of these 7 tumor autoantigens in the diagnosis of LC, and the diagnostic AUCs are all around 0.5–0.7 [3, 25, 26]. However, there are certain differences in sensitivity and specificity. For example, Ouyang et al. [8] found that the sensitivity of combined detection in diagnosing LC was 44.02% and the specificity was 83%. In the selected population, Mu et al. [27] found that the sensitivity and specificity of combined diagnosis were 25.42% and 91.75%, respectively. We found that the sensitivity and specificity of combined detection were 86.14% and 48.02%, respectively. We believe that the differences in the sensitivity and specificity of this combined detection for diagnosing LC may be related to differences in the included population, geographical differences, different degrees of progression of LC patients, and detection methods.

This study also had some limitations. First, key informative elements of the clinical data we collected were lacking, such as traditional risk factors associated with lung cancer, such as smoking and alcohol consumption, and no stratified studies were conducted for subjects with different baseline data. Differences in autoantibody levels in LC patients with different clinical progression could not be further captured. Second, we did not obtain data on patients with benign nodules. In addition, prognostic data on lung cancer patients were also unavailable due to the difficulty of follow-up.

## 6. Conclusion

Through our research, it can be found that the detection of seven-autoantibody of LC alone and combined detection have certain value in the diagnosis of LC in Yunnan. The combined detection of these seven-autoantibody can be considered as an indicator for early screening and diagnosis of LC to make up for the low sensitivity of traditional tumor markers to early LC.

## Figures and Tables

**Figure 1:** The experimental procedure of this study.

**Figure 2:** Receiver operating curves (ROC) for the detection of seven-autoantibody alone and in combination in the diagnosis of LC. (a) ROC of serum anti-CAGE for the diagnosis of LC. (b) ROC of serum Anti-GAGE7 for the diagnosis of LC. (c) ROC of serum anti-GBU4-5 in the diagnosis of LC. (d) ROC of serum anti-MAGE A1 in the diagnosis of LC. (e) ROC of serum anti-P53 in the diagnosis of LC. (f) ROC of serum anti-PGP9.5 in the diagnosis of LC. (g) ROC of serum anti-SOX2 in the diagnosis of LC. (h) ROC of combined detection of serum anti-CAGE, anti-GAGE7, anti-GBU4-5, anti-MAGE A1, anti-P53, anti-PGP9.5, and anti-SOX2 in the diagnosis of LC.

**Figure 3:** Combined detection of serum anti-CAGE, anti-GAGE7, anti-GBU4-5, anti-MAGE A1, anti-P53, anti-PGP9.5, and anti-SOX2 for the diagnosis of different histological types of LC. (a) Combined detection of serum anti-CAGE, anti-GAGE7, anti-GBU4-5, anti-MAGE A1, anti-P53, anti-PGP9.5, and anti-SOX2 for the diagnosis of squamous cell carcinoma. (b) Combined detection of serum anti-CAGE, anti-GAGE7, anti-GBU4-5, anti-MAGE A1, anti-P53, anti-PGP9.5, and anti-SOX2 for the diagnosis of adenocarcinoma. (c) Combined detection of serum anti-CAGE, anti-GAGE7, anti-GBU4-5, anti-MAGE A1, anti-P53, anti-PGP9.5, and anti-SOX2 for the diagnosis of small cell lung cancer.

**Table 1:** Comparison of clinical data between LC patients and control groups.

	LC (*N* = 329)	Controls (*N* = 202)	Statistical value	*P* value
Age (year)	49.49 ± 12.03	50.65 ± 12.51	1.063	0.288

Sex				
Male	155	105	1.187	0.276
Female	174	97		

Histological type				
Squamous cell carcinoma	125	—		
Adenocarcinoma	143	—		
Small cell lung cancer	61	—		

TNM staging				
I	89	—		
II	95	—		
III	73	—		
IV	72	—		

**Table 2:** Comparison of serum levels of seven-autoantibody in LC patients and control groups.

	LC (*N* = 329)	Controls (*N* = 202)	*U*-value	*P* value
Anti-CAGE (U/mL)	0.10(0.10, 0.50)	0.10(0.10, 0.23)	−3.630	<0.001
Anti-GAGE7 (U/mL)	1.40(0.60, 2.80)	0.80(0.40, 1.60)	−4.633	<0.001
Anti-GBU4-5 (U/mL)	0.70(0.10, 2.30)	0.50(0.10, 1.40)	−2.721	<0.001
Anti-MAGE A1 (U/mL)	0.40(0.20, 1.00)	0.30(0.10, 0.60)	−4.365	<0.001
Anti-P53 (U/mL)	1.40(0.60, 2.80)	1.10(0.50, 2.50)	−2.343	0.019
Anti-PGP9.5 (U/mL)	0.70(0.20, 1.80)	0.20(0.18, 0.63)	−6.528	<0.001
Anti-SOX2 (U/mL)	0.80(0.30, 2.60)	0.50(0.20, 1.60)	−3.371	0.001

**Table 3:** Evaluation of the diagnostic value of serum seven-autoantibody alone and in combination for LC.

	AUC (95% CI)	*P* value	Sensitivity (%)	Specificity (%)	Cut-off value
Anti-CAGE	0.586(0.537–0.634)	<0.001	98.02	16.41	1.850 U/mL
Anti-GAGE7	0.620(0.572–0.667)	<0.001	67.33	52.28	1.350 U/mL
Anti-GBU4-5	0.570(0.521–0.619)	0.007	96.53	15.50	5.050 U/mL
Anti-MAGE A1	0.612(0.563–0.660)	<0.001	68.32	47.42	0.150 U/mL
Anti-P53	0.561(0.510–0.611)	0.019	46.53	64.44	0.950 U/mL
Anti-PGP9.5	0.667(0.619–0.715)	<0.001	55.94	71.43	0.250 U/mL
Anti-SOX2	0.587(0.538–0.636)	<0.001	54.46	60.79	0.550 U/mL
Combined factor	0.719(0.676–0.761)	<0.001	86.14	48.02	—

## Data Availability

All data supporting this study are available from the corresponding author.
